# Efficacy of Fenestration Decompression for the Treatment of Oral and Maxillofacial Cysts

This article has been retracted.

**DOI:** 10.1155/2022/2262547

**Published:** 2022-06-28

**Authors:** Zhangyi Li

**Affiliations:** Department of Stomatology, The Fifth Central Hospital of Tianjin, Tianjin 300450, China

## Abstract

**Background:**

Surgery is the mainstay of treatment for oral and maxillofacial cysts. Compared with open surgery that will bring more harm to patients, fenestration decompression, as a surgical method with good curative effects and little damage, has received increasing attention in the treatment of oral and maxillofacial cysts.

**Methods:**

The clinical data of 135 patients with oral and maxillofacial cysts visited the Fifth Central Hospital of Tianjin between June 2019 and September 2021 were collected for retrospective analysis. Patients were assigned to two groups based on the treatment plan implemented: the control group (*n* = 64) treated with curettage of cysts and the observation group (*n* = 71) with fenestration decompression. Therapeutic efficacy parameters and surgical indicators were detected. Additionally, postoperative cyst, pain, complication rate, and recurrence, as well as life quality six months after treatment, were evaluated and compared.

**Results:**

In comparison with the control group, the observation group was observed to have a higher total effective rate, less operation time, shorter hospital stays, and less intraoperative bleeding (*P* < 0.05). In addition, the shrinkage rate, shrinkage volume, and postoperative density of the cyst cavity were higher in the observation group than in the control group (*P* < 0.05). The observation group also outperformed the control group with lower postoperative VAS score, complication rate, and half-year recurrence rate (*P* < 0.05). Furthermore, significantly better life quality was determined in the observation group after half a year of treatment (*P* < 0.05).

**Conclusion:**

Fenestration decompression is highly effective in treating oral and maxillofacial cysts, contributing to fewer complications, markedly relieved symptoms, shorter hospitalization time, well-preserved facial nerves, and low recurrence rate in the later period, which is worthy of clinical promotion.

## 1. Introduction

Oral and maxillofacial cysts (OMC) are a relatively common type of diseases requiring oral and maxillofacial surgery, the main lesions of which comprise hard and soft tissue cysts. Hard tissue cysts are mainly divided into keratinizing cysts and radicular cysts, while soft tissue cysts include submandibular gland cysts, sublingual gland cysts, and epidermoid cysts [1, 2]. The clinical symptoms of OMC are not so obvious at early stage that they are easily ignored by patients, often leading to the worsening of the condition when seeking medical treatment. In addition, the occurrence of certain tissue structure damage, such as keratinizing cysts and apical cysts, will bring greater challenges to clinical treatment [3, 4]. Without prompt and effective treatment, there will be secondary infections, suppuration, swelling, and pain, seriously affecting patients' daily life [5].

Surgery, a common treatment for OMC, has been shown to be helpful to the recovery of patients. Although there are many effective surgical options for OMC, a unified treatment plan has yet to be determined, with great controversies on the one with the best effect and highest safety [6]. In the past clinical practice, open surgeries, such as jawbone resection and cyst curettage, were often used for the treatment of OMC, bringing great damage to patients' teeth, blood vessels, and physical condition with slow wound recovery [7]. In addition, the economic burden resulting from slow postoperative recovery can also directly affect the life quality of patients and their families [8]. Therefore, it is extremely important to find a surgical approach with less trauma and better curative effects. With the advances in science and technology in clinical treatment, fenestration decompression (FD) has opened a new chapter in OMC treatment, attracting widespread attention [9].

Herein, 135 patients were selected, some of whom were treated with FD and were observed in terms of clinical efficacy, postoperative complications, recurrence, etc., providing references for OMC treatment as well as the clinical application of FD in treating the disease.

## 2. Materials and Methods

### 2.1. Clinical Information

In this retrospective study, we gathered the clinical data from 135 patients with OMC presented to the Fifth Central Hospital of Tianjin between June 2019 and September 2021. Patients were assigned to two groups based on the treatment plan they received: the control group (*n* = 64) treated with curettage of cysts and the observation group (*n* = 71) with FD. Inclusion criteria were as follows: (1) presence of with oral and maxillofacial cysts [10], (2) in accordance with the surgical indications, (3) good oral condition and healthy periodontal tissue, (4) compliance with the doctor's orders to complete oral hygiene and cleaning, (5) and complete clinical data. Exclusion criteria were as follows:: (1) pregnant and lactating women, (2) alcoholic fatty liver disease and/or various types of viral hepatitis, (3) serious cardiocerebrovascular and blood system diseases, (4) organic mental disorders, (5) high risk of malignancy in cysts, and (6) incomplete clinical data and refusing to participate in the study. This research has been approved by the Ethics Committee of the Fifth Central Hospital of Tianjin and was conducted in compliance with the Declaration of Helsinki. All patients signed informed consent for participation.

### 2.2. Treatment Methods

Cyst curettage was performed in the control group, specifically as follows: under CT and X-ray display, the location, size, and correlation of the patient's oral and maxillofacial cysts with surrounding tissues were determined. After local anesthesia, an incision was made in the patient's oral cavity, and the weak bone area of the jaw was cut open to fully expose and completely remove the cyst. The bone cavity was then treated with iodine tincture. After the bleeding was completely stopped, a rubber drainage column was placed, and the wound was closed and sutured, followed by postoperative anti-inflammatory and swelling treatment.

FD was performed in the observation group, specifically as follows: the operation was performed under local anesthesia. After incising a 1 cm × 1.5 cm mucoperiosteal flap at the most bulging and weakest part of the oral vestibular cyst, the mucoperiosteum was peeled off to remove exposed thin tissue with an osteotome or rongeur. The bone fragments were then removed to expose the cyst wall, and the cyst wall tissue of the same size was cut for pathological examination. Next, the cystic cavity was examined, and a curved vascular clamp was used to extend into the cystic cavity and pierce the possible septum. Cystic cavity was thoroughly flushed with normal saline, followed by tamponade with iodoform gauze for drainage. One week later, the drainage iodoform gauze was removed, the cyst cavity was rinsed, and the cyst plug was inserted into the fenestration to keep the wound from healing and keep the drainage port open. After the operation, the patient's mouth was rinsed with normal saline before and after meals, and the surgical incision was properly treated with anti-inflammatory hemostasis and detumescence drugs until the patient recovered and was discharged from the hospital. Both groups of patients were followed up for half a year by means of outpatient service, home visits, and telephone visits, with their postoperative complications and cyst recurrence recorded.

### 2.3. Observation Indexes

(1) Therapeutic efficacy, mainly divided into markedly effective, effective, and ineffective shown by CT and X-ray results, was assessed and compared. Markedly effective was as follows: the patient's facial cyst tissue was completely eliminated without residue, and the incision healed well. Effective was as follows: the patient's facial cyst tissue was basically eliminated with a small amount of residues, and the incision could be healed. Ineffective was as follows: most of the patient's facial cyst tissue remained, with unsatisfactory incision healing and even infections: total effective rate = (markedly effective + effective) cases/total number of cases × 100%. (2) Surgical indexes (operation time, hospitalization time, intraoperative blood loss) were also recorded and compared. (3) Postoperative cyst conditions of two groups were recorded and compared, including cyst cavity shrinkage rate, cyst cavity shrinkage volume, and postoperative cyst cavity density. (4) The Visual Analogue Scale (VAS) [11], with the total score being 10 points and the score positively related to the pain, was used to evaluate and compare the postoperative pain between the two groups. (5) We also recorded postoperative complications, including alveolar nerve injury, bone defect, tooth defect, and postoperative infection, for comparison. (6) The recurrence of cysts was recorded during the 6-month follow-up performed on all patients. (7) Assessment of patients' quality of life before and half a year after treatment was conducted using the Short-Form 36 Item Health Survey (SF-36) [12]. The total score was 100 points, and higher scores suggest a better quality of life

### 2.4. Statistical Processing

Statistical analysis and plotting of the data collected employed SPSS 19.0 (IBM) and GraphPad 7, respectively. Count data, described as percentages, were statistically analyzed by the chi-square test. For the comparison of measurement data between groups, the Student *t*-test was used. *P* < 0.05 was supposed to indicate a statistically significant difference.

## 3. Results

### 3.1. Comparison of General Information

As indicated by Table 1, the two groups had no significant differences regarding gender, age, and body mass index (BMI), indicating compatibility of the enrolled subjects (*P* > 0.05).

### 3.2. Comparison of Clinical Therapeutic Effects

The number of cases with markedly effective, effective, and ineffective treatment in the observation group was 40, 29, and 2, respectively, with an overall effective rate of 97.18%. While the corresponding data in the control group was 20, 31, and 13, respectively, the total effective rate was 79.69%. The above data showed a significantly higher treatment effective rate in the observation group compared with the control group (*P* < 0.05, Table 2).

### 3.3. Comparison of Surgical Indicators

The comparison of surgical indicators (Table 3) showed that the observation group had statistically shorter operation time and length of hospital stay and less intraoperative blood loss than the control group (*P* < 0.05).

### 3.4. Comparison of Postoperative Cysts

After treatment, the shrinkage rate, shrinkage volume, and postoperative density of the cyst cavity were found to be higher in the observation group as compared to the control group (*P* < 0.05, Table 4).

### 3.5. Comparison of Postoperative Pain

A statistically lower postoperative VAS score was determined in the observation group when compared to the control group (*P* < 0.05, Figure 1).

### 3.6. Comparison of Postoperative Complications

After statistical analysis (Table 5), it was found that the incidence of complications was lower in the observation group (5.63%) than in the control group (23.44%) (*P* < 0.05).

### 3.7. Comparison of Recurrence

During the 6-month follow-up, relapse was observed in 2 cases in the observation group and 17 cases in the control group, presenting a statistically lower recurrence rate in the observation group (2.82%) compared with the control group (26.56%) (*P* < 0.05, Table 6).

### 3.8. Comparison of Quality of Life before and after Treatment

The SF-36 scores of both groups increased statistically after treatment (*P* < 0.05). Moreover, the observation group had a higher SF-36 score (95.98 ± 2.49 points) than the control group (90.63 ± 2.02 points) (*P* < 0.05, Figure 2).

## 4. Discussion

OMC, a kind of common clinical disease, is mainly attributed to the proliferation of oral epithelium and epithelial cells, followed by the formation of liquefied cyst lesions, progression of cystic lesions, swelling of cysts, and displacement of corresponding tissues, which impair facial functions to varying degrees [13]. In recent years, the incidence of OMC shows an upward trend with the continuous progress of material life and the change of dietary structure [14]. The diseased part of OMC is relatively special with slow growth and is often spherical with clear boundaries and a soft, doughy feel to the touch. Patients generally have nonspecific symptoms in the initial stage, while in the middle and late stages, cysts may expand and cause severe damage to the jaw tissue if left untreated. Moreover, teeth in the affected area may become loose and fall off, directly affecting the patient's facial appearance, oral health, and normal chewing function and even causing facial deformities and cancer that affect patient's quality of life to a great extent [15]. Therefore, early detection, diagnosis, and treatment are necessary to effectively improve the prognosis of patients.

The clinical treatment of OMC mainly includes jawbone resection, cyst curettage, and chemical treatment, which can eliminate cysts to a certain extent. However, most of the above methods are invasive that will bring trauma to the patient's oral cavity with a high incidence of complications, making them difficult to meet the expectations of clinical treatment and patients [16]. As modern medical technology advances, the concept of minimally invasive surgery has been broadly accepted and applied in various clinical departments. Studies have pointed out that FD for OMC has the advantages of low complication rate and favorable treatment efficacy [17]. However, there is still a lack of comprehensive curative effect analysis of FD in OMC, which was further explored in the present study. Our findings demonstrated that FD can achieve better therapeutic effects than open surgery for the treatment of OMC, with higher total effective rate observed and recorded in the observation group. FD is a surgical procedure in which the local cyst wall is incised and drained in the most damaged area of the jawbone. It can effectively reduce the intracystic pressure, eliminate the hypertonic state in the cyst, and block the way the cyst fluid absorbs water, thereby achieving the purpose of eliminating cysts [18]. Meanwhile, the internal and external pressure of the cyst is in a state of equilibrium under FD, allowing the gradual repair and reconstruction of the surrounding bone, thereby preserving the integrity of the jaw [19]. With the reduction of damage to the jawbone and effective removal of cystic tissue, the clinical treatment effect can be effectively ensured. It was also found in our study that, compared to the control group, the observation group showed significantly less operation time, hospitalization time and intraoperative bleeding, and lower postoperative VAS scores, all suggesting that the application of FD in OMC patients contributes to obviously better related indexes and relieved postoperative pain of patients. It is mainly because the surgical operation of FD is simpler compared to conventional open surgery, without the need for external incision for cyst tissue curettage; so, the time required for the operation is greatly shortened [20]. In addition, the incision of FD is smaller and will not cause trauma to the patient's jaw, which can not only reduce the amount of intraoperative blood loss but also alleviate postoperative pain and speed up postoperative recovery to a certain extent [21]. FD has been conducted in the treatment of degenerative lumbar spinal stenosis. It was found that FD could effectively reduce intraoperative blood loss and postoperative drainage and relieve low back pain in patients as suggested by the short-term follow-up [22]. In addition, the postoperative complication and recurrence rates were compared, and the results identified markedly lower indexes in the observation group, indicating that FD can further reduce postoperative complications among OMC patients. As a surgery that incises and drains the cyst tissue, FD does not cause major damage to the patient's oral cavity during the operation, which is conducive to reducing the occurrence of bone defect, tooth defect, alveolar nerve injury, and postoperative infection [23]. Finally, we compared patients' quality of life and found an obviously better quality of life in the observation group after six months of treatment, suggesting that FD has a significant effect on improving patients' postoperative life quality.

## 5. Conclusion

To sum up, FD is highly effective in the treatment of OMC, contributing to fewer complications, markedly relieved clinical symptoms, shorter hospitalization time, well preserved facial nerves, and lower recurrence rate, which reserves clinical popularization. This study also has some deficiencies. Because of limited samples and short research period of this study, the research results have certain contingency. Therefore, further research is needed to obtain more scientific data on the application effect of FD in OMC patients. We will further carry out multicenter and large-sample studies to provide more convincing data to refine and support our research results.

## Figures and Tables

**Figure 1:** Comparison of postoperative pain between two groups of patients. Note: ^∗^ indicates *P* < 0.05.

**Figure 2:** Comparison of life quality before and after treatment. Note: ^∗^ indicates *P* < 0.05.

**Table 1:** Comparison of general information.

Factors	Observation group (*n* = 71)	Control group (*n* = 64)	*t*/*χ*^2^	*P*
Gender			0.568	0.451
Male	39 (54.93)	31 (48.44)		
Female	32 (45.07)	33 (51.56)		
Age (years)			0.038	0.848
≥42	30 (42.25)	26 (40.63)		
<42	41 (57.75)	38 (59.38)		
BMI (kg/m^2^)			0.001	0.921
≥23	35 (49.30)	31 (48.44)		
<23	36 (50.70)	33 (51.56)		
Disease duration (years)	1.62 ± 0.33	1.68 ± 0.28	1.133	0.259
History of smoking			0.116	0.733
Yes	42 (59.15)	36 (56.25)		
No	29 (40.85)	28 (43.75)		
History of drinking			0.369	0.543
Yes	37 (52.11)	30 (46.88)		
No	34 (47.89)	34 (53.13)		
Level of education			0.165	0.684
Junior high school and below	26 (36.62)	21 (32.81)		
Junior high school and above	45 (63.38)	43 (67.19)		

**Table 2:** Comparison of clinical therapeutic effects.

Items	Observation group (*n* = 71)	Control group (*n* = 64)	*χ* ^2^	*P*
Markedly effective	40 (56.34)	20 (31.25)	—	—
Effective	29 (40.85)	31 (48.44)	—	—
Ineffective	2 (2.82)	13 (20.31)	—	—
Effective rate of treatment	69 (97.18)	51 (79.69)	10.43	0.001

**Table 3:** Comparison of surgical indicators.

Items	Observation group (*n* = 71)	Control group (*n* = 64)	*χ* ^2^	*P*
Operation time (min)	52.93 ± 2.12	81.95 ± 3.21	62.54	<0.001
Intraoperative blood loss (ml)	97.6 ± 3.05	158.47 ± 5.38	81.87	<0.001
Length of hospital stay (d)	5.18 ± 0.3	8.16 ± 0.33	54.96	<0.001

**Table 4:** Comparison of postoperative cysts.

Indexes	Observation group (*n* = 71)	Control group (*n* = 64)	*χ* ^2^	*P*
Cyst shrinkage rate (%)	84.04 ± 2.14	62.21 ± 2.6	53.36	<0.001
Cyst shrinkage volume (mm^2^)	52.23 ± 2.09	36.41 ± 1.1	54.16	<0.001
Postoperative cyst density (g/m^2^)	0.53 ± 0.08	0.34 ± 0.07	14.61	<0.001

**Table 5:** Comparison of postoperative complications.

Indexes	Observation group (*n* = 71)	Control group (*n* = 64)	*χ* ^2^	*P*
Bone defect	1 (1.41)	4 (6.25)	—	—
Tooth defect	2 (2.82)	3 (4.69)	—	—
Alveolar nerve injury	1 (1.41)	3 (4.69)		
Postoperative infection	1 (1.41)	5 (7.81)	—	—
Complication rate	4 (5.63)	15 (23.44)	8.822	0.003

**Table 6:** Comparison of recurrence.

Recurrence	Observation group (*n* = 71)	Control group (*n* = 64)	*χ* ^2^	*P*
Number of cases with recurrence	2	17	15.69	<0.001
Rate of recurrence	2.82%	26.56%		

## Data Availability

The labeled dataset used to support the findings of this study are available from the corresponding author upon request.
